The article "COQ10B Knockdown Modulates Cell Proliferation, Invasion, Migration, and Apoptosis in Esophageal Squamous Cell Carcinoma" was retracted in 2023. Reasons: unreliable results or conclusions; lack of ethics approval or compliance; concerns about the data; concerns about the peer review.

# COQ10B Knockdown Modulates Cell Proliferation, Invasion, Migration, and Apoptosis in Esophageal Squamous Cell Carcinoma

**DOI:** 10.1155/2022/6247824

**Published:** 2022-07-21

**Authors:** Yu Wei, Juan Liu, Yan Gao, Xiaoli Ma, Leiyu Cao, Nuersimanguli Maimaitiming, Chengcheng Qu, Li Zhang

**Affiliations:** Department 4 of Comprehensive Internal Medicine of Healthy Care Center for Cadres, The First Affiliated Hospital of Xinjiang Medical University, Urumqi, Xinjiang Uygur Autonomous Region, China

## Abstract

**Objective:**

Esophageal squamous-cell carcinoma (ESCC) is an aggressive malignant tumor, accounting for more than 90% of esophageal cancers. However, treatments such as surgical resection, radiotherapy, and chemotherapy are unable to achieve ideal clinical outcomes. The purpose of this study was to explore the effects of COQ10B on proliferation, apoptosis, migration, and invasion of esophageal squamous-cell carcinoma (ESCC) cells.

**Methods:**

Quantitative real-time PCR (qRT-PCR) was used to detect the expression of COQ10B in ESCC and normal tissues and in ESCC cell lines (KYSE-150 and TE-1). MTT assay and flow cytometry were applied to investigate the effects of COQ10B shRNA lentivirus (LV-shCOQ10B) on ESCC cell proliferation and apoptosis, respectively. The effect of COQ10B silencing on ESCC cell migration and invasion was determined by wound healing assay and transwell invasion assay, respectively.

**Results:**

The expression of COQ10B mRNA in ESCC tissues was higher than that in surrounding tissues. The decreased COQ10B level in KYSE-150 and TE-1 cells by LV-shCOQ10B could inhibit cell proliferation, promote cell apoptosis, and reduce the ability of invasion and migration (all *P* < 0.05).

**Conclusion:**

COQ10B was highly expressed in human ESCC tissues. COQ10B silencing contributed to the inhibition of proliferation, invasion, and migration of ESCC cells and the promotion of cell apoptosis, suggesting COQ10B may be a potential molecular target for the diagnosis and treatment of ESCC.

## 1. Introduction

Esophageal cancer is one of the most common gastrointestinal malignancies, and the incidence and the mortality of esophageal cancer, respectively, rank eighth and sixth worldwide according to Global Cancer Statistics in 2021 [1]. It was estimated that its 5-year survival was less than 20% [2]. In China, esophageal cancer is a leading cause of death, rating number four of all cancers, which results in huge burden of public health [3]. Esophageal squamous-cell carcinoma (ESCC) is induced by the malignant transformation of esophageal epithelial cells and has unique epidemiological and pathophysiological characteristics [4]. ESCC is one of the main subtypes of esophageal malignant tumors, which is responsible for more than 90% of esophageal cancers. It is more prevalent in Asia, East Africa, and South America [5]. Although advances had been improved in the diagnosis and treatment technology of ESCC, the 5-year overall survival rate remains 15–20% [6]. Clinical prognosis of ESCC is highly associated with the stage at the time of diagnosis. Estimated 5-year survival for ESCC patients with local disease, regional disease, and distant metastasis was 45.2%, 23.6%, and 4.8%, respectively [4]. In view of the atypical early symptoms of patients with ESCC and lack of early diagnosis technique, 70%–80% of patients diagnosed in the middle and late stage have lost the opportunity of operation, and most of them are treated with comprehensive treatment such as radiotherapy and chemotherapy [7,8]. At present, the pathogenesis of ESCC remains to be explored. Therefore, in-depth elucidation of the molecular mechanism of ESCC occurrence and development is of great importance for accurate diagnosis and treatment of ESCC, contributing to prognosis improvement and mortality decrease.

The article "COQ10B Knockdown Modulates Cell Proliferation, Invasion, Migration, and Apoptosis in Esophageal Squamous Cell Carcinoma" was retracted in 2023. Reasons: unreliable results or conclusions; lack of ethics approval or compliance; concerns about the data; concerns about the peer review.

Coenzyme Q10 (COQ10, also known as ubiquinone [9]) as a putative steroidogenic acute regulatory protein-related lipid transfer domain protein participated in the oxidation reaction of respiratory chain in mitochondria, thus enhancing the synthesis of adenosine triphosphate (ATP) in mitochondria [10, 11]. As reported, diseases such as neurodegenerative diseases, fibromyalgia, diabetes, cancer, mitochondrial diseases, muscular diseases, and heart failure are associated with decreased circulating levels of CoQ10 [12], which could be transformed into reducing substance with antioxidant activity to be involved in regulation of cell characteristics [13, 14]. The dysregulated expression of COQ10B (Ensembl: ENSG00000115520; NCBI GeneID: 80219; GenBank accession: NM_025147, genomic location: 2q33.1; size: 238 amino acids) (https://www.genecards.org/cgi-bin/carddisp.pl?gene=COQ10B), an isoform of COQ10 [14], has been detected in chronic stress-associated intestinal barrier dysfunction [15], acute pelvic inflammatory illness [16], moyamoya disease [17], and pelvic inflammatory disease [16]. However, the role of COQ10B in tumor progression has not been widely reported. Therefore, we attempted to investigate COQ10B expression in ESCC, as well as its effect on cell proliferation, apoptosis, invasion, and migration of ESCC cells *in vitro*.

## 2. Materials and Methods

### 2.1. Sample Collection

Forty samples of esophageal squamous-cell carcinoma (ESCC) and the surrounding tissues (3–5 cm away from the edge of cancer lesion) after tumor resection were collected in the First Affiliated Hospital of Xinjiang Medical University from January 2021 to December 2021, which were all preserved in liquid nitrogen for COQ10B gene expression. All the included patients did not receive radiotherapy, chemotherapy, or other anti-tumor treatment prior to operation.

The article "COQ10B Knockdown Modulates Cell Proliferation, Invasion, Migration, and Apoptosis in Esophageal Squamous Cell Carcinoma" was retracted in 2023. Reasons: unreliable results or conclusions; lack of ethics approval or compliance; concerns about the data; concerns about the peer review.

### 2.2. Cell Culture

ESCC lines, including KYSE-150 and TE-1 (Shanghai Genechem Co., Ltd., China), were cultured in RPMI1640 medium with 10% fetal bovine serum (FBS) (Ausbian, Australia), 100 u/ml penicillin, and 100 *μ*g/ml streptomycin in an incubator with 5% CO_2_ at 37°C. Het-1A, a human normal esophagus epithelial cell (ATCC, China), was cultured in BEGM medium in the atmosphere of 95% air and 5% CO_2_ at 37°C.

### 2.3. Construction of COQ10B shRNA Lentivirus (LV-shCOQ10B)

Design of RNA interference target was performed prior to synthetize single-stranded DNA oligo (Shanghai Generay Biotech Co., Ltd., China) containing interference sequence and annealing pairing for generation of double-stranded DNA, followed by connection of lentivirus vector GV115 digested with enzymes through restriction sites at the two ends of DNA. The ligation product was transferred to prepared TOP 10 competent cell of *Escherichia coli*. The positive recombinants were identified by PCR and then verified by sequencing. The plasmids were extracted following correct clones from the sequencing results.

### 2.4. COQ10B shRNA Lentivirus Transduction

The KYSE-150 and TE-1 cells were divided into LV-shCOQ10B group and LV-shCtrl group, which were infected with LV-shCOQ10B and control shRNA lentivirus, respectively. In brief, the target cells were plated in 12-well plate 24 hours prior to viral infection, which were added with 1 ml of complete optimal medium (with serum and antibiotics) overnight. The cells were approximately 80% confluent on the day of infection. In the case of lentivirus infection labeled by fluorescence, the expression of GFP was observed under the fluorescence microscope according to the infection time point determined in the pre-experiment.

### 2.5. Quantitative Real-Time PCR (qRT-PCR) Detection

Extraction of total RNAs from tissues and cell lines was conducted by TRIzol reagents, followed by the measurement of their concentration and purity. Synthesis of cDNA was performed by reverse transcriptase kits (RIBOBIO, China). The amplification of cDNA was carried out with PCR kits (RIBOBIO, China) on ABI7500 platform. The primer sequences are listed in Table 1, and the relative expression level of COQ10B was determined by the 2^−ΔΔCt^ method using GAPDH as internal reference.

### 2.6. 3-[4, 5-Dimethylthiazol-2-yl]-2, 5 Diphenyl Tetrazolium Bromide (MTT)

KYSE-150 and TE-1 cells in logarithmic phase of growth were, respectively, seeded in 96-well plate with 2000 per well and cultured in an incubator containing 5% CO_2_ at 37°C, followed by additional culture with 20 *μ*l MTT reagent (5 mg/ml) (Genview, USA) for 4 h, and then 2–5 min oscillation was operated with the supplement of 150 *μ*l DMSO in the absence of supernatant. The optical density (OD) with a 490 nm filter was detected by microplate reader using reagents (New England Biolabs, USA). Cell growth curve was obtained with time as abscissa and OD value as ordinate.

The article "COQ10B Knockdown Modulates Cell Proliferation, Invasion, Migration, and Apoptosis in Esophageal Squamous Cell Carcinoma" was retracted in 2023. Reasons: unreliable results or conclusions; lack of ethics approval or compliance; concerns about the data; concerns about the peer review.

### 2.7. Flow Cytometry Assay

Flow cytometer (Millipore, USA) was used to evaluate ESCC cell apoptosis. KYSE-150 and TE-1 infected cells in logarithmic phase of growth were detached by trypsin (Sangon Biotech (Shanghai) Co., Ltd., China) and resuspended in medium. The cell suspension was centrifugated at 1300 rpm for 5 min. D-Hanks precooled at 4°C was carried to wash the cells in absence of supernatant. Bling buffer was applied to additional cell washing and the cells were stained with 10 *μ*l Annexin V-APC, followed by analysis of number of cell apoptosis at different stages by guava InCyte software.

### 2.8. Wound Healing Assay

KYSE-150 and TE-1 cells (4 × 10^4^ cells/well) were placed into 96-well plate overnight. After changing a low concentration serum medium, the cell reaching more than 90% of cell confluence was scratched with instrument. The scratches were observed by fluorescence microscope after rinsed with serum-free medium for 2-3 times in 5% CO_2_ at 37°C. Migration area at three time points (0 h and 24 h) was analyzed by Celigo.

### 2.9. Transwell Invasion Assay

After 48 h infection, KYSE-150 and TE-1 cells (1 × 10^5^ cells/well) were, respectively, resuspended with 500 *μ*L serum-free medium. The cell suspension was put into the upper chamber of transwell (8 *μ*m pore size) (Corning, USA) treated with matrigel matrix, and 750 *μ*L medium with 10% FBS was added to the lower chamber. The cells with additional 20 h incubation migrated to the bottom were fixed with methanol and stained with 0.1% Giemsa. The images were captured under microscope (×200).

### 2.10. Western Blot

The total protein of KYSE-150 and TE-1 cells was extracted and quantified by BCA reagents according to the instructions. Total protein (50 *μ*g) was separated by sodium dodecyl sulfate-polyacrylamide gel electrophoresis (SDS-PAGE), followed by being transferred to the polyvinylidene difluoride (PVDF) membrane. After blocking with 5% non-fat milk, the following antibodies were added overnight at 4°C, including anti-Akt antibody (1 : 1000) and p-Akt antibody (1 : 1000). The PVDF membrane was rinsed with TBST buffer for 15 min for 3 times and then probed with HRPO goat anti-mouse IgG-HRP and Goat anti-Rabbit IgG-HRP for 1 h incubation. After washing of PVDF membrane by BST buffer for 15 min for 3 times, immunoblots were revealed by Alpha imaging system.

The article "COQ10B Knockdown Modulates Cell Proliferation, Invasion, Migration, and Apoptosis in Esophageal Squamous Cell Carcinoma" was retracted in 2023. Reasons: unreliable results or conclusions; lack of ethics approval or compliance; concerns about the data; concerns about the peer review.

### 2.11. Statistical Analysis

Data analysis was performed by SPSS 25.0 software, and graphics were constructed by GraphPad Prism 8.0 software. All data were expressed as mean ± standard deviation. Independent sample *t*-test is used for the comparison between the two groups, and the one-way ANOVA is applied to the comparison between multiple groups followed by Tukey's HSD test. *P* < 0.05 indicated that the difference was statistically significant.

## 3. Results

### 3.1. Overexpression of COQ10B in ESCC

In order to investigate COQ10B expression in ESCC, we collected tumor and surrounding tissues from 40 ESCC patients for qRT-PCR detection, and the result revealed the higher expression of COQ10B in ESCC tissues than that in surrounding normal tissues (1.644 ± 0.543 vs. 0.793 ± 0.492, *P* < 0.05, Figure 1(a)). *In vitro,* the relative mRNA expression of COQ10B in ESCC cell lines (KYSE-150 and TE-1) were increased as compared with human normal esophagus epithelial Het-1A cell (Figure 1(b)). Therefore, KYSE-150 and TE-1 cells were selected as follow-up experiments.

### 3.2. Efficacy of COQ10B shRNA Lentivirus Transduction in ESCC Cells

To ensure the efficacy of COQ10B shRNA lentivirus transduction in ESCC cells (KYSE-150 and TE-1 cells), it was observed under fluorescence microscope, and the results demonstrated the efficiency of >80% (Figure 2(a)). Furthermore, lentivirus efficiency was also validated by performing qRT-PCR, which revealed LV-shCOQ10B decreased COQ10B mRNA in KYSE-150 and TE-1 cells as compared with those treated with LV-shCtrl (*P* < 0.05, Figure 2(b)). Therefore, using LV-shCOQ10B to knock down COQ10B was preferable for the subsequent experiments.

### 3.3. COQ10B Knockdown Could Inhibit Malignant Biological Characteristics of ESCC Cells

To find the effect of COQ10B silencing on ESCC cell proliferation and cell cycle, detections of MTT assay and flow cytometry were performed. As illustrated in Figures 3–5, LV-shCOQ10B suppressed the cell proliferation of KYSE-150 and TE-1 cells, arrested the cells in *S* phrase, and increased cell apoptosis. Moreover, the wound healing assay and transwell assay were used to determine the migration and invasion of ESCC cells, which were suppressed in KYSE-150 and TE-1 cells after infected with COQ10B shRNA lentivirus (Figures 6 and 7). All mentioned above indicated that COQ10B knockdown could inhibit malignant biological characteristics of ESCC cells.

The article "COQ10B Knockdown Modulates Cell Proliferation, Invasion, Migration, and Apoptosis in Esophageal Squamous Cell Carcinoma" was retracted in 2023. Reasons: unreliable results or conclusions; lack of ethics approval or compliance; concerns about the data; concerns about the peer review.

### 3.4. PI3K/AKT Pathway May Be Involved in KYSE-150 Cells after COQ10B Silencing

To find the possible involvement of PI3K/AKT pathway in ESCC cells after COQ10B silencing, the assessment of western blot revealed a significant reduced expression of AKT and p-AKT protein expression in LV-shCOQ10B group as compared to the LV-shCtrl group (Figure 8), revealing the regulation role of COQ10B in KYSE-150 cells via PI3K/AKT signaling pathway.

## 4. Discussion

At present, the treatments for ESCC are surgical resection, radiotherapy, and chemotherapy. However, these treatments are unable to achieve ideal clinical outcomes, leading to severe challenges in prognosis evaluation of ESCC [18]. Therefore, exploring molecules related to prognosis has important guiding significance for the intervention of patients with ESCC.

In non-tumor diseases, such as diabetes, kidney disease, and inflammation, COQ10 affects cell metabolism concerning cell transport, transcriptional regulation, and cell signal transduction [19, 20]. The association between COQ10 and tumors has been reported. For example, Jolliet et al. [21] indicated that increased COQ10 levels in plasma of patients with breast cancer were associated with good prognosis. However, supplementation with CoQ10 reduced some of the important markers of inflammation and MMPs in patients with breast cancer [22]. Meanwhile, CoQ10 showed a tendency to be associated with improved prognosis of lung cancer [23]. Recently, few evidences of subtype *A* or *B* affecting tumor progression have been found. COQ10B as a subtype of COQ10 may have different function. Therefore, in-depth studies targeting the role of COQ10B in regulation of ESCC are necessary. In this study, qRT-PCR detection revealed highly expressed COQ10B in human ESCC tissues and cell lines as compared with normal tissues and cells, respectively, suggesting that COQ10B as a oncogene may be associated with the occurrence and development of ESCC.

Next, we cultured ESCC cell lines (KYSE-150 and TE-1) for COQ10B shRNA lentivirus transduction to knockdown COQ10B, which result in significantly decreased proliferation and promoted apoptosis of KYSE-150 and TE-1 cells. These data showed that COQ10B expression was highly associated with ESCC cell proliferation and apoptosis, and the overexpression of COQ10B may be an important factor for the increased malignancy of ESCC cells. The accurate transition from G1 phase of the cell cycle to S phase is crucial for the control of cell proliferation, and its misregulation promotes oncogenesis [24]. Furthermore, increased KYSE-150 and TE-1 cells in S phase were observed after COQ10B knockdown with the decreased cells in G1 phase.

The article "COQ10B Knockdown Modulates Cell Proliferation, Invasion, Migration, and Apoptosis in Esophageal Squamous Cell Carcinoma" was retracted in 2023. Reasons: unreliable results or conclusions; lack of ethics approval or compliance; concerns about the data; concerns about the peer review.

Cell migration is an essential process in physiological and pathological phenomena such as embryonic development, angiogenesis, wound healing, immune response, inflammatory response, and atherosclerosis and is also an essential step in tumor metastasis [25–27]. In this study, cell migration ability was weakened in LV-shCOQ10B group compared to the LV-shCtrl group, indirectly indicating that COQ10B promoted ESCC cell migration and enhanced risk of distant metastasis. Cell invasion refers to the ability of tumor cells, with the help of their own motility, to penetrate the original tissue and reach the surrounding and distant sites [28]. We conducted transwell invasion assay to mimic the tumor cell invasion environment, and the results showed that KYSE-150 and TE-1 cells with decreased COQ10B (LV-shCOQ10B group) exhibited a diminished ability to traverse the chambers as compared to LV-shCtrl group. These evidences revealed that COQ10B was estimated to promote ESCC cell invasion which acts as a typical characteristic of tumor malignant biology.

Phosphatidylinositol-4, 5-bisphosphate 3-kinase (PI3K) is activated by numerous genes and leads to the binding of Akt to cell membrane through phosphoinositide dependent kinase in PI3K/AKT signal transduction pathway [29]. PI3K/AKT signaling pathway is involved in multiple biological processes of tumor pathogenesis [30, 31], including cellular energy metabolism, cell proliferation, apoptosis, and angiogenesis [29, 32, 33]. In a previous study, CoQ10 activated the downstream PI3K/AKT signaling pathway, thus resulting in wound closure in human immortalized keratinocyte HaCaT cells [34]. Besides, CoQ10 augments rosuvastatin neuroprotective effect in a model of global ischemia via the activation of AKT signaling pathway [35], which also restores A*β*_25–35_ oligomer-inhibited proliferation of neural stem cells (NSCs) by activating the PI3K/AKT pathway [36]. Our study performed western blot to determine the expression of PI3K/AKT signaling pathway related proteins. It was found that COQ10B silencing inhibited the expression levels of Akt and p-AKT proteins in ESCC cells, demonstrating that COQ10B may be involved in the regulation of PI3K/AKT signaling pathway.

Our study had some limitations. Firstly, our limited sample sizes may lead to the bias of our results, and more experiments are required to confirm it. Secondly, the protein expression of COQ10B in ESCC tissues would be detected using immunohistochemical staining or western blotting although its level had been examined *in vitro*. Thirdly, the relationship between COQ10B expression and clinical factors would be further explored deeply. Fourthly, at least two shRNA sequences for COQ10B would be used to avoid a possibility of off-target effects. Finally, the *in vivo* experiment is not performed due to time and funding constraints, which would be explored in the future to validate the *in vitro* results.

The article "COQ10B Knockdown Modulates Cell Proliferation, Invasion, Migration, and Apoptosis in Esophageal Squamous Cell Carcinoma" was retracted in 2023. Reasons: unreliable results or conclusions; lack of ethics approval or compliance; concerns about the data; concerns about the peer review.

To sum up, COQ10B was upregulated in ESCC tissues and cells. COQ10B silencing contributed to the inhibition of cell proliferation, promotion of cell apoptosis, and decreased invasion and migration ability of ESCC cells. COQ10B may be used as a vital biomarker and therapeutic target molecule of esophageal cancer for further research.

## Figures and Tables

**Figure 1:** The relative expression level of COQ10B in ESCC. Note: the qRT-PCR was used to determine the relative expression level of COQ10B in ESCC tissues and normal tissues (surrounding non-cancerous tissues) ((a, ^*∗*^*P* < 0.05), a well as in ESCC (KYSE-150 and TE-1) and human normal esophagus epithelial cell (Het-1A) (b); ∗ indicates ^*∗*^*P* < 0.05 compared with Het-1A cell.

**Figure 2:** Lentivirus-mediated COQ10B knockdown in KYSE-150 and TE-1 cells. (a) Representative microscopic images of KYSE-150 and TE-1 cells infected with recombinant lentivirus expressing green fluorescence. (b) Lentivirus-mediated COQ10B knockdown in KYSE-150 and TE-1 cells, verified by qRT-PCR. ^*∗*^*P* < 0.05.

**Figure 3:** MTT detection for cell proliferation of KYSE-150 and TE-1 cells after lentivirus-mediated COQ10B knockdown. ^*∗*^*P* < 0.05.

**Figure 4:** Flow cytometric analysis of cell cycle of KYSE-150 and TE-1 cells after lentivirus-mediated COQ10B knockdown. ^*∗*^*P* < 0.05.

**Figure 5:** Flow cytometric analysis of cell apoptosis of KYSE-150 and TE-1 cells after lentivirus-mediated COQ10B knockdown. ^*∗*^*P* < 0.05.

**Figure 6:** The width of scratch area from 0 h to 24 h of KYSE-150 and TE-1 cells after lentivirus-mediated COQ10B knockdown. ^*∗*^*P* < 0.05.

**Figure 7:** Representative view and statistics of KYSE-150 and TE-1 cells transferring from the apical chamber of the transwell system coated with matrigel into the basolateral chamber after lentivirus-mediated COQ10B knockdown. ^*∗*^*P* < 0.05.

**Figure 8:** The protein levels of PI3K/AKT signal pathway related factors in KYSE-150 cells after lentivirus-mediated COQ10B knockdown.

**Table 1:** Primer sequences for qRT-PCR.

Gene	Primer sequence
COQ10B	Forward: 5′-TGGAGACTATTTGGCGTTTTAGC-3′
	Reverse: 5′-GCAAGCTGGGAATGTAGAAGTG-3′
GAPDH	Forward: 5′-TGACTTCAACAGCGACACCCA-3′
	Reverse: 5′-CACCCTGTTGCTGTAGCCAAA-3′

## Data Availability

The data used to support the findings of this study are included within the article.
